# Cord Blood Stem Cell-Mediated Induction of Apoptosis in Glioma Downregulates X-Linked Inhibitor of Apoptosis Protein (XIAP)

**DOI:** 10.1371/journal.pone.0011813

**Published:** 2010-07-28

**Authors:** Venkata Ramesh Dasari, Kiran Kumar Velpula, Kiranpreet Kaur, Daniel Fassett, Jeffrey D. Klopfenstein, Dzung H. Dinh, Meena Gujrati, Jasti S. Rao

**Affiliations:** 1 Department of Cancer Biology and Pharmacology, University of Illinois College of Medicine at Peoria, Peoria, Illinois, United States of America; 2 Department of Neurosurgery, University of Illinois College of Medicine at Peoria, Peoria, Illinois, United States of America; 3 Department of Pathology, University of Illinois College of Medicine at Peoria, Peoria, Illinois, United States of America; Universidade de São Paulo, Brazil

## Abstract

**Background:**

XIAP (X-linked inhibitor of apoptosis protein) is one of the most important members of the apoptosis inhibitor family. XIAP is upregulated in various malignancies, including human glioblastoma. It promotes invasion, metastasis, growth and survival of malignant cells. We hypothesized that downregulation of XIAP by human umbilical cord blood mesenchymal stem cells (hUCBSC) in glioma cells would cause them to undergo apoptotic death.

**Methodology/Principal Findings:**

We observed the effect of hUCBSC on two malignant glioma cell lines (SNB19 and U251) and two glioma xenograft cell lines (4910 and 5310). In co-cultures of glioma cells with hUCBSC, proliferation of glioma cells was significantly inhibited. This is associated with increased cytotoxicity of glioma cells, which led to glioma cell death. Stem cells induced apoptosis in glioma cells, which was evaluated by TUNEL assay, FACS analyses and immunoblotting. The induction of apoptosis is associated with inhibition of XIAP in co-cultures of hUCBSC. Similar results were obtained by the treatment of glioma cells with shRNA to downregulate XIAP (siXIAP). Downregulation of XIAP resulted in activation of caspase-3 and caspase-9 to trigger apoptosis in glioma cells. Apoptosis is characterized by the loss of mitochondrial membrane potential and upregulation of mitochondrial apoptotic proteins Bax and Bad. Cell death of glioma cells was marked by downregulation of Akt and phospho-Akt molecules. We observed similar results under *in vivo* conditions in U251- and 5310-injected nude mice brains, which were treated with hUCBSC. Under *in vivo* conditions, Smac/DIABLO was found to be colocalized in the nucleus, showing that hUCBSC induced apoptosis is mediated by inhibition of XIAP and activation of Smac/DIABLO.

**Conclusions/Significance:**

Our results indicate that downregulation of XIAP by hUCBSC treatment induces apoptosis, which led to the death of the glioma cells and xenograft cells. This study demonstrates the therapeutic potential of XIAP and hUCBSC to treat malignant gliomas.

## Introduction

Apoptosis is the cell's intrinsic death program that controls normal tissue homeostasis. Apoptosis pathways can be initiated through death receptors or mitochondria and usually result in activation of caspases as common effector molecules [1]. Evasion of apoptosis is one of the hallmarks of human cancers, including glioblastoma [2]. One mechanism through which tumor cells are believed to acquire resistance to apoptosis is by overexpression of XIAP (X-linked inhibitor of apoptosis protein). XIAP has received interest as a therapeutic target as it is probably the IAP member best characterized with respect to structure and biochemical mechanism [3]–[5]. XIAP interacts with and inhibits active caspases-3, -7 and -9 [6]–[8]. Recent studies confirmed that overexpression of XIAP confers resistance to multi-agent chemotherapy, including stimuli of the mitochondrial and death receptor pathways of caspase activation [9]–[11]. Through its ability to inhibit caspases, overexpression of XIAP renders cells resistant to multi-agent chemotherapy. XIAP is frequently overexpressed in malignant cells and, in certain patients, is associated with poor clinical outcome [12]. Knocking out XIAP with siRNA or antisense oligonucleotides restores chemosensitivity to a variety of malignant cell lines [13]–[16]. Characterization of XIAP-deficient mice proved that knocking out XIAP is not toxic to normal cells as evidenced by a lack of significant pathology in the XIAP knockout mouse [17]. However, there have been very few reports of the downregulation of XIAP in human glioblastoma cells.

Human umbilical cord blood is an alternative source of adult stem cells. Several reports indicate that human umbilical cord blood derived mesenchymal stem cells (hUCBSC) are similar to stem cells from bone marrow with respect to cell characteristics and multilineage differentiation potential [18]–[20]. Recently, hUCBSC were proved to be more advantageous in cell procurement, storage, and transplantation than bone marrow–derived mesenchymal stem cells [21]. These hUCBSC were used to induce cytotoxicity in malignant glioma cells [22] and to show their migration capacity towards glioma cells [23]. Under *in vivo* conditions, TRAIL-secreting hUCBSC were used against intracranial gliomas [24]. However, the mechanistic aspects of hUCBSC against apoptosis induction in glioma have not been well established.

Hence, in the present study, we investigated the effects of both hUCBSC and siXIAP (shRNA for XIAP) in the downregulation of XIAP and thus inducing apoptosis in glioblastoma cells both *in vitro* and *in vivo*. We observed that downregulation of XIAP in glioma cells induced apoptosis involving mitochondria. This has been correlated with mitochondrial membrane potential damage and inhibition of survival and proliferation of glioma cells. In addition, we evaluated the *in vivo* effects of hUCBSC against glioma xenografts for the induction of apoptosis and pathway specific proteins.

## Results

### Co-culture of glioma cells with hUCBSC downregulates XIAP

For all the experiments of this study we used hUCBSC which are positive for CD29 and CD81 (data not shown). To evaluate the efficiency of hUCBSC, we tested the effect of hUCBSC on glioma cells in co-cultures for 3 days. In order to make sure that inhibition of cell proliferation, induced cytotoxicity, observed apoptotic phenotype and decreased protein expressions of XIAP and Akt in glioma cells, the co-cultures were grown in the same media which was used for growing glioma cells alone, as described in Materials and Methods. We performed MTT assay and cytosolic LDH cytotoxicity assays to study the effect of hUCBSC on the glioma cells. We observed that hUCBSC inhibited proliferation of the glioma cell lines and the inhibition was more than 50% in all the cell lines tested (Fig. 1A). Also, cytotoxicity induced by hUCBSC was significant (*p*<0.05) and more than 50% in all the cell lines (Fig. 1B). Xenograft cell lines 5310 and 4910 were found to have more cytotoxicity than glioma cell lines SNB19 and U251. We next tested whether or not this cytotoxicity resulted in the cell death or not. For this, we ran FACS analyses of all the single and co-cultures of cell lines using Annexin V. All the glioma cell lines in co-culture with hUCBSC were found to have more than 50% apoptotic cells (Fig. 1C). In order to check the expression of apoptotic proteins, we ran immunoblot analysis of XIAP, Akt and pAkt molecules, which are highly upregulated in glioma cells. As expected, XIAP was highly downregulated in all the co-cultures of glioma cells (Fig. 1D). The downregulation of XIAP was correlated with the downregulation of Akt and pAkt^S473^. As a control experiment to evaluate the effect of hUCBSC on glioma cells, we co-cultured glioma cells with normal human astrocytes and observed the effect of astrocytes on glioma cells. Astrocytes did not show any effect on the status of XIAP, Akt and phospho-Akt in the glioma cells (Fig. 1E). These results suggest that hUCBSC are efficiently inducing cytotoxicity and apoptosis in order to inhibit proliferation of glioma cells by way of downregulating XIAP and phosphorylated form of Akt. To confirm that downregulation of XIAP results in the inhibition of phosphorylation of Akt, the glioma cells were transfected with shRNA of XIAP (siXIAP). In all four of the cell lines, siXIAP inhibited proliferation (Fig. S1A), induced cytotoxicity (Fig. S1B), and induced apoptosis in a significant manner (*p*<0.05) (Fig. S1C). We routinely checked for the expression of XIAP in cells transfected with siXIAP; XIAP was highly silenced resulting in the decrease in the phosphorylation of Akt in cells treated with siXIAP as compared to scrambled vector (SV) (Fig. S2). These results confirm that co-culture with hUCBSC and siXIAP treatment of glioma cells inhibits growth and proliferation of glioma cells by inducing cytotoxicity and apoptosis by downregulating XIAP. Further, to evaluate the process of apoptosis, we performed TUNEL analysis of the cells co-cultured with hUCBSC or treated with siXIAP. Both these treatments induced significant apoptosis in glioma cells (*p*<0.05) (Fig. 2A) as compared to control and SV treatments. However, when compared to hUCBSC treatments, siXIAP treatments induced apoptosis in greater number of cells (Figs. 2B and 2C). In order to confirm the time period at which hUCBSC show their effect on glioma cells, we did time-course experiments. Glioma cells were co-cultured with hUCBSC at different time periods (24 h, 48 h and 72 h) and the cell lysates were analyzed by immunoblot analysis. In both U251 and 5310 cell lines of the present study, 72 h period was found to be more effective in inhibiting XIAP and Akt and inducing apoptosis in glioma cells (Fig. S3).

**Figure 1:** Growth inhibition of glioma cells by hUCBSC. (A) MTT assay of single and co-cultures of glioma cells with hUCBSC. Even though proliferation values of both single cultures of glioma cells and hUCBSC were taken as 100%, values of proliferation of glioma + hUCBSC cocultures were calculated in relation to single cultures of glioma alone. When we calculated values of proliferation of glioma + hUCBSC cocultures in relation to single cultures of hUCBSC, we got much less values compared to the values presented here. (B) Cytotoxicity assay based on cytosolic LDH assay. (C) FACS analysis results of glioma cells showing apoptotic cells as measured by Annexin V. Immunoblot analysis of proteins showing expression of XIAP, Akt and pAkt^Ser473^ in (D) single and co-cultures of glioma cells with hUCBSC and (E) single and co-cultures of glioma cells with astrocytes. 40 µg of proteins were loaded onto 12% gels and transferred onto nitrocellulose membranes and probed with respective antibodies. Immunoreactive bands were visualized using chemiluminescence ECL Western blotting detection reagents and the reaction was detected using Hyperfilm-MP autoradiography film. Each experiment was repeated 3 times. Error bars indicate ±SEM. * Significant at *p*<0.05.

**Figure 2 pone-0011813-g002:** Evaluation of apoptosis of glioma cells by TUNEL assay. (A) Single and co-cultures of glioma cells and hUCBSC and siXIAP-transfected glioma cells were seeded in 8-well chamber slides. After various treatments, TUNEL assay was done using *in situ* cell death detection kit (Roche) as per the manufacturer's protocol. (B) Quantitative estimation of TUNEL cells in hUCBSC treatments. (C) Quantitative estimation of TUNEL cells in siXIAP treatments. Each experiment was repeated 3 times. The results show a significant increase in the number of apoptotic cells with siXIAP and hUCBSC treatments as compared to the control and SV treatments. Inset pictures show DAPI. SV = scrambled vector. n = 3. * Significant at *p*<0.05.

To identify the molecular mechanisms that underlie the induced apoptosis in glioma cells treated with hUCBSC and siXIAP, we focused on the Bcl-2 family of apoptosis regulators that integrate cellular survival and apoptotic signals through their action on mitochondria. We reasoned that both hUCBSC and siXIAP might activate pro-apoptotic members of the Bcl-2 family (e.g., Bax) in order to allow the glioma cells to undergo apoptosis. For this, we assessed immunoblots of pro-apoptotic proteins Bax and Bad. Both Bax and Bad proteins were highly upregulated and associated with a decrease in the expression of Bcl-2 protein in hUCBSC treatments compared to single cultures of glioma cells (Fig. 3A). Similar results were observed in siXIAP treatments compared to control and SV treatments (Fig. S2). These results confirm that in both the treatments, Bax and Bad were highly upregulated, thereby confirming the involvement of mitochondria during apoptotic induction. Increasing evidence suggests that altered mitochondrial function is linked to apoptosis, and a decreasing mitochondrial transmembrane potential is associated with mitochondrial dysfunction [25]. Hence, we tested whether upregulation of Bax and Bad is correlated with damage to mitochondrial membrane potential in these glioma cells. In hUCBSC treatments, SNB19 cells showed the highest percentage (84.17%) of mitochondrial membrane potential damage followed by 5310 (59.33%), 4910 (59.19%) and U251 (58.68%) (Fig. 3B). On the other hand, in siXIAP treatments, the highest mitochondrial membrane potential damage was observed in 4910 (71.91%) followed by 5310 (71.67%), U251 (66.96%) and SNB19 (64.28%) (Fig. 3C). These results confirm that the hUCBSC and siXIAP treatments induced upregulation of Bax and Bad to involve mitochondria in apoptosis, and this is significantly associated with mitochondrial membrane potential damage in all the glioma cells used in this study. These results are in agreement with our hypothesis that co-cultures of glioma cells with hUCBSC induced apoptosis involving mitochondria, ultimately leading to death of the glioma cells, and the action of hUCBSC is similar to silencing of XIAP.

**Figure 3 pone-0011813-g003:** Downregulation of XIAP induces mitochondrial apoptosis. Immunoblot analysis of proteins showing expression of (A) Bax, Bad and Bcl-2 in co-cultures of glioma cells with hUCBSC treatments. 40 µg of proteins were loaded onto 14% gels, transferred onto nitrocellulose membranes and probed with respective antibodies. Immunoreactive bands were visualized using chemiluminescence ECL Western blotting detection reagents and the reaction was detected using Hyperfilm-MP autoradiography film. Mitochondrial membrane potential damage was evaluated using Mitotracker red (Invitrogen). (B) Shows mitochondrial membrane potential damage in co-cultures and (C) in siXIAP treatments. Each experiment was repeated 3 times. SV = scrambled vector. Error bars indicate ±SEM. * significant at p<0.05.

Further, we evaluated whether or not downregulation of XIAP in glioma cells activates the caspase enzymes leading to apoptosis. We measured caspase-3 activity in glioma cells alone and in co-culture with hUCBSC. Co-culture of hUCBSC activated caspase-3 enzyme in a significant manner in the glioma cells (*p*<0.05) (Fig. 4A). For this assay, we also used human astrocytes alone and in co-culture with hUCBSC. Contrary to glioma cells, hUCBSC did not activate caspases in astrocytes. In a similar way, we also tested the activity of caspase-9 since this enzyme is related to mitochondrial apoptosis. Co-cultures of hUCBSC with glioma cells show higher activity of caspase-9 whereas hUCBSC did not induce any activity of caspase-9 in astrocytes (Fig. 4B). The efficiency of these analyses was checked by the application of inhibitors of caspase-3 and caspase-9 which showed reduced levels of caspases. These results show that induction of apoptosis by hUCBSC is exclusive to glioma cells only but not to normal cells such as astrocytes. We also tested the siXIAP treatments for inducing the activity of caspases and observed that both caspase-3 and caspase-9 are activated by siXIAP treatments (Fig. S4). Further, to evaluate the effect of hUCBSC on glioma cells and normal astrocytes, we tested the expression of pAkt (S^473^) in the cell lysates by immunoblot analyses. Expression of pAkt in U251 and 5310 cells was downregulated by hUCBSC in co-cultures whereas in astrocytes, there was no effect on the expression pAkt (Fig. 4C). However, Akt inhibitor IV downregulated phosphorylation of Akt in all 3 cell lines U251, 5310 and astrocytes. In another experiment, we used Akt inhibitor IV for 30′ to inhibit phosphorylation of Akt in U251, 5310 and astrocytes and then co-cultured them with hUCBSC for 3 days. In both glioma cell lines U251 and 5310, pAkt levels were downregulated whereas in astrocytes, they were brought back to the normal levels. That means, even though Akt inhibitor IV inhibited the phosphorylation of Akt in astrocytes, co-culture with hUCBSC restored the phosphorylation status of Akt in astrocytes alone. These results confirm that inhibition of phosphorylation of Akt by hUCBSC is exclusively restricted to only the glioma cells but not to normal astrocytes. Rather, normal cells are restored to normal phosphorylation levels of Akt by hUCBSC to enhance their growth and proliferation. These results confirm our previous observations with cortical neurons, where we have shown that cord blood stem cells protect cortical neurons against glutamate toxicity following Akt pathway (56).

**Figure 4:** Activity of caspases in single and co-cultures of cells. (A) Caspase-3 activity in single and co-cultures of hUCBSC with glioma cells or human astrocytes. (B) Caspase-9 activity in single and co-cultures of hUCBSC with glioma cells or human astrocytes. Both of these assays were done as described in Materials and Methods. C3I =  Caspase-3 Inhibitor (Ac-DEVD-CHO); C9I =  Caspase-9 inhibitor (Ac-LEHD-CHO). Each experiment was repeated 3 times. Error bars indicate ±SEM. * Significant at *p*<0.05. (C) Cell lysates of the respective treatments were immunoblotted and probed with pAkt (S^473^) and respective GAPDH. Akt inhibitor IV was used at a concentration of 10 µM per ml for 30′ at 37°C and 5% CO_2_ in an incubator (n = 3).

### Downregulation of XIAP by hUCBSC treatment has an anti-tumor effect in U251 and 5310 glioma nude mice models

Our *in vitro* experiments have proven that co-cultures with hUCBSC can efficiently inhibit glioma cell proliferation, causing cytotoxicity and leading to apoptosis. Therefore, we further investigated the anti-tumor effect of these stem cells *in vivo* using U251 and 5310 cells in nude mice. After the mice were implanted with U251, 5310 and hUCBSC as explained in Materials and Methods, the mice were observed for 21 days. At that point, tumor samples were taken, and paraffin-embedded sections were prepared for immunohistopathological examination. Hematoxylin and Eosin (H&E) staining of the *in vivo* sections clearly showed that the tumors in hUCBSC-treated mice were inhibited significantly and were one-third of the size of the tumors in control mice brains (*p*<0.05) (Figs. 5A and 5B). Then, we checked for the induction of apoptosis in hUCBSC-treated tumors by TUNEL assay. Sections of nude mice brains treated with hUCBSC clearly show the presence of more numbers of TUNEL cells indicating that the tumor cells are undergoing apoptosis (Fig. 5C). Next, we evaluated XIAP expression in nude mice brain tissue lysates by immunoblotting. The tissue lysates showed significant reduction of XIAP, Akt and pAkt in hUCBSC-treated mice tumors (*p*<0.05) (Fig. 5D). Quantitation of Western bands revealed that XIAP and pAkt were significantly downregulated in hUCBSC treatments compared to control tumors (Fig. 5E). Also, we ran reverse-transcription based PCR to check the expression of XIAP in control tumor and hUCBSC-treated tumor brain samples. In both the hUCBSC-treated xenograft brains, XIAP levels were highly downregulated (Fig. 5F). We further evaluated the expression of XIAP mRNA by means of FISH analysis. Control tumor brain sections of both U251 and 5310, which were probed with anti-sense XIAP oligonucleotides, showed higher expression of XIAP mRNA (Fig. 5G). Compared to these, hUCBSC-treated brain sections showed very low expression of XIAP mRNA, proving the fact that hUCBSC downregulate XIAP under *in vivo* conditions. These results confirm our *in vitro* experiments that hUCBSC downregulate XIAP in the glioma cells.

**Figure 5:** Induction of apoptosis in nude mice brain tumors by hUCBSC *in vivo*. Nude mice with pre-established intracranial human glioma tumors (U251 or 5310) were treated with hUCBSC by intracranial injection (2×10^5^). Fourteen days after hUCBSC administration, the brains were harvested, sectioned, and stained with Hematoxylin and Eosin (n = 3). Bar  = 500 µm. (A) Inhibition of intracranial tumors by hUCBSC *in vivo*. (B) Quantification of tumor size (n≥3). Error bars indicate ±SEM. * Significant at *p*<0.05. (C) TUNEL analysis of control and hUCBSC treated sections. Bar  = 200 µm. Immunoblot analysis of proteins showing expression of (D) XIAP, Akt and pAkt in tissue lysates of brains. (E) Quantitative estimation of (D). 40 µg of proteins were loaded onto 12% gels and transferred onto nitrocellulose membranes and probed with respective antibodies. Immunoreactive bands were visualized using chemiluminescence ECL Western blotting detection reagents and the reaction was detected using Hyperfilm-MP autoradiography film. Error bars indicate ±SEM. * Significant at *p*<0.05. (F) Reverse-transcription based PCR was run using cDNA from control and tumor and hUCBSC-treated tumor brains and using XIAP and β-actin primers. (G) Detection of XIAP in nude mice brain sections by Fluorescent in situ hybridization (FISH) analysis: Control and hUCBSC treated sections were processed for FISH analysis as explained in Materials and Methods. Bar  = 200 µm.

In order to evaluate the mechanism by which apoptosis is induced in the nude mice tumor brains, we carried out immunohistochemistry on brain sections with cleaved caspase-3 antibody. Since XIAP is downregulated in the mice tumors, we hypothesized that caspases should be active in these tumor sections. As expected, caspase-3 was highly expressed in hUCBSC-treated sections (Fig. 6A). We further evaluated the tissue lysates using immunoblot analysis and observed that TNF-α, TRAIL and cleaved PARP are highly upregulated in hUCBSC treatments (Fig. 6B). In stem cell treatments, both caspase-3 and TNF-α were significantly upregulated compared to control tumor brains (*p*<0.05) (Fig. 6C). These results confirm that downregulation of XIAP in mice tumor brains induces the activation of caspase-3, which induced apoptosis. In both *in vitro* and *in vivo* experiments we observed that the process of apoptosis was induced by the activation of death ligand TRAIL (Fig. S2, Fig. S3 and Fig. 6). Together, all these apoptotic proteins are involved in the cleavage of PARP in the nucleus, thereby leading to cell death. Finally, we checked whether mitochondria were involved in the process of apoptosis in the mice tumor brains similar to the *in vitro* results. We probed the tumor sections as well as hUCBSC-treated sections with Bax antibody. We carried out co-localization studies with CD81 (a mesenchymal stem cell marker for hUCBSC) and Bax antibodies. In hUCBSC-treated sections, Bax is highly upregulated when compared to the control tumor brains. Further, Bax was co-localized with CD81, confirming the presence of hUCBSC in treated brains (Fig. 6D). These results were confirmed by immunoblot analysis of Bax and Bad proteins in tissue lysates, which showed highly elevated levels in the treated samples (Fig. 6E). Quantification of Western bands shows that both Bax and Bad were significantly upregulated in stem cell treatments compared to control tumor sections (*p*<0.05) (Fig. 6F). Finally, we tested the involvement of Smac/DIABLO in the induction of apoptosis by hUCBSC. We performed co-localization experiments with Smac/DIABLO and MTCO2 in the brain sections of both treated and untreated samples. In control tumor brain sections, Smac/DIABLO was co-localized in the mitochondria whereas in hUCBSC-treated brain sections, Smac/DIABLO was co-localized in the nucleus (Fig. 7). These results show that mitochondrial apoptosis was involved in the hUCBSC-treated tumors. Taken together, these results confirm the anti-tumor effect of hUCBSC *in vivo* and that glioma cell apoptosis *in vitro* is efficiently induced by hUCBSC by the downregulation of XIAP.

**Figure 6:** Upregulation of caspase-3 and Bax in nude mice brains. Nude mice with pre-established intracranial human glioma tumors (U251 or 5310) were treated with hUCBSC by intracranial injection (2×10^5^). Fourteen days after hUCBSC administration, the brains were harvested, sectioned and immunoprobed for caspase 3 using appropriate HRP-conjugated secondary antibody. (A) Expression of cleaved caspase-3 activity in brain sections. Bar  = 200 µm. (B) Immunoblot analysis of proteins showing expression of cleaved caspase 3, TNF-alpha, TRAIL and cleaved PARP in tissue lysates of brains. (C) Quantitative estimation of (B). 40 µg of proteins were loaded onto 12–14% gels and transferred onto nitrocellulose membranes and probed with respective antibodies. Immunoreactive bands were visualized using chemiluminescence ECL Western blotting detection reagents and the reaction was detected using Hyperfilm-MP autoradiography film. (D) *In vivo* expression of Bax. Brain sections were immunoprobed for Bax and CD81 using appropriate secondary antibodies. Bax is labeled with Alexa Fluor-594 conjugated secondary antibody and CD81 is labeled with Alexa Fluor-488 conjugated secondary antibody. Bar  = 200 µm. (E) Immunoblot analysis of proteins showing expression of Bax and Bad in tissue lysates of brains. 40 µg of proteins were loaded onto 14% gels and transferred onto nitrocellulose membranes and probed with respective antibodies. Immunoreactive bands were visualized using chemiluminescence ECL Western blotting detection reagents and the reaction was detected using Hyperfilm-MP autoradiography film. (F) Quantitative estimation of (E).

**Figure 7:** Co-localization of Smac/DIABLO in treated and untreated brain tumors. Nude mice with pre-established intracranial human glioma tumors (U251 or 5310) were treated with hUCBSC by intracranial injection (2×10^5^). Fourteen days after hUCBSC administration, the brains were harvested, sectioned and immunoprobed for Smac/DIABLO (second mitochondria-derived activator of caspase/direct IAP binding protein with low PI) and MTCO2 (Mitochondrial Cytochrome Oxidase subunit 2 – mitochondrial marker) using appropriate HRP-conjugated secondary antibodies. Smac/DIABLO is Alexa Fluor-488 conjugated and MTCO2 is Alexa Fluor-594 conjugated. Bar  = 200 µm.

## Discussion

Malignant gliomas are the most commonly diagnosed malignant adult primary brain tumors. Resistance to induction of cell death by apoptosis in response to radiotherapy or chemotherapy is one of the hallmarks of many solid tumors, including glioblastoma. These tumors overexpress XIAP. The principle mechanism underlying the anti-apoptotic activity of XIAP has been proposed to be direct caspase inhibition [26]. Many reports in cultured cells have demonstrated that overexpression of XIAP confers resistance to multi-agent chemotherapy, including stimuli of the mitochondrial and death receptor pathways of caspase activation [9]–[11]. Knocking out XIAP with siRNA or antisense oligonucleotides restores chemosensitivity to a variety of malignant cell lines [13]–[16]. Finally, knocking out XIAP is not toxic to normal cells, as evidenced by a lack of significant pathology in the XIAP knockout mouse [17]. Hence, in this study, we used hUCBSC as well as siXIAP to downregulate XIAP, thereby inducing apoptosis in glioma cells.

Co-culturing of glioma cells with hUCBSC resulted in the loss of XIAP protein and the induction of cell death in the absence of external death stimuli (Figs. 1–[Fig pone-0011813-g002] [Fig pone-0011813-g003] 4), illustrating an essential survival function of XIAP in glioma cells. In a similar manner, siRNA for XIAP induced death in the absence of external death stimuli to glioma cells. We observed that the depletion of XIAP led to the activation and processing of caspases and the activation of Bad and Bax proteins in the mitochondria to induce apoptosis. This is further correlated with the downregulation of Akt and pAkt molecules. Akt is overactivated in many glioblastomas due to the loss of PTEN function [27], [28]. Akt regulates the function of numerous downstream signaling proteins involved in cell cycle, proliferation, apoptosis and invasion, which are all important to tumorigenesis [29]. Activated Akt deregulates cell growth by stabilization of cyclin D and promotion of the nuclear entry of mdm2, leading to the degradation of p53 [30]. On the other hand, activated Akt exerts anti-apoptotic activity by phosphorylating and inactivating pro-apoptotic signaling proteins, such as Bad and caspase-9 [29], [31]. Akt is one of the anti-apoptotic factors that must be activated through phosphorylation. The involvement of Akt in diverse tumorigenic activities suggests that Akt activation alone might be sufficient to induce cancer [32].

In this study, XIAP downregulation is correlated with the downregulation of Akt in both the treatments, suggesting that these treatments inhibit the activation of Akt, which inhibits the growth and survival of glioma cells. Recently, it was proposed that XIAP acts as an E3 ubiquitin ligase for PTEN and promotes Akt activity by regulating PTEN content and compartmentalization [33]. In accordance with this report, previously we have shown that hUCBSC upregulated PTEN while downregulating XIAP [59]. Our present results are in accordance with the previous reports, and downregulation of XIAP did result in the downregulation of Akt and inhibition of glioma cell growth, while inducing apoptosis.

An alternative mechanism mediating XIAP-dependent protection from apoptosis involves transcriptional activity mediated via the stimulation of NF-κB, which depends on the E3 ubiquitin ligase activity of the RING domain of XIAP [34]. NF-κB is composed of two subunits, p65relA and p50, which are members of the REL protein family. There are different pathways by which NF-κB can be activated; cytokines such as tumor necrosis factor-α (TNF-α) activate their receptor, and in turn recruit the complex of inhibitor of κB (IκB) kinase (IKK), resulting in IKK phosphorylation. IKK kinases include members of the mitogen-activated protein kinase (MAPK) family, such as NF-κB-inducing kinase (NIK) [35]. In the present study, we observed that hUCBSC upregulated TNF-α in the mice brains, suggesting that hUCBSC simultaneously activates both the NF-κB-activated and caspase-mediated apoptotic pathways. Recently, it was shown that TRAIL kills malignant glioma cells through induction of apoptosis, providing a new therapeutic strategy for these tumors [36]–[38]. It was suggested that TRAIL may induce activation of intrinsic mitochondrial pathways, which may amplify and rescue TRAIL receptor-mediated caspase 8-initiated activation of the caspase cascade in the extrinsic pathway [37]. Local delivery of soluble TRAIL [39], TRAIL-expressing adenoviral vector [24] and TRAIL-secreting neural stem cells [40] have all been shown to induce apoptosis in intracranial gliomas. Systemic administration of soluble TRAIL along with chemotherapeutic drugs inhibits glioma growth without causing neurological impairment or damage to normal tissue in mice [41]. Our study shows that, in glioma cells as well as in nude mice brain tumors, hUCBSC induced TRAIL activation, which ultimately resulted in the induction of apoptosis.

It has been demonstrated that induction of apoptosis requires involvement of the Bcl-2 family including apoptosis inhibiting gene products (e.g., Bcl-2, Bcl-XL) and apoptosis accelerating gene products (e.g., Bad, Bax, Bak, Bcl-XS, Bim) [42], [43]. The susceptibility of tumor cells to induction of apoptosis is controlled by the ratio between pro-apoptotic and anti-apoptotic proteins such as Bax/Bcl-2 [44]. It has been reported that Bax is associated with apoptotic cell death [45], [46]. During apoptosis, Bax is translocated to the mitochondria where it promotes the release of proteins from the intermembrane space into cytoplasm, an important step in apoptosis. Bax also interacts with the permeability transition pore to facilitate protein movement through the mitochondrial membrane [25], [47], [48]. Our results indicate a critical role of XIAP in modulating the ratio of Bcl-2/Bax and increased Bax protein expression in mediating apoptosis in glioma cells. These changes ultimately led to the activation of downstream caspases (caspases-9 and -3) and eliciting an apoptosis response. In the present study, in both *in vitro* and *in vivo* systems, hUCBSC increased Bax and Bad expression. Thus, induction of apoptosis by hUCBSC involves Bax and Bad, which explains the role of mitochondria in cell death. A decrease in mitochondrial membrane potential plays an important role in cell death [49]–[51]. However, the role of mitochondrial membrane potential in cell death induced by stem cells remains unclear. In the present study, both hUCBSC and siXIAP treatments caused significant reduction in mitochondrial membrane potential before the induction of cell death. This might result in mitochondrial depolarization through the inhibition of respiratory chain [52]. Our results clearly establish inhibition of XIAP functions as a potential way to sensitize glioma cells to apoptosis.

Since XIAP inhibits both initiator and effector caspases, in the present study hUCBSC downregulated XIAP which resulted in the activation of caspases. Caspases play a key role during the execution phase in various forms of apoptosis [53]. To evaluate the role of caspase activation in the hUCBSC-induced cell death of glioma cells, the effect of caspase inhibitors on hUCBSC-induced cell death was examined. In this report, we demonstrated that hUCBSC induced the activation of both caspase-9 and caspase-3. Activation of the caspase-9/Apaf-1/cytochrome c apoptosome in the mitochondrial-dependent apoptotic pathway leads, in turn, to caspase-3 activation [54]. Hence, it is plausible that during the induction of apoptosis by hUCBSC, mitochondrial upregulated Bax and Bad induce the activation of caspase-9 in glioma cells which ultimately triggers the activation of caspase-3, ultimately leading to the apoptotic death by the cleavage of PARP. Here, we have demonstrated that this particular induction of the activity of caspases is restricted to glioma cells only and not to normal cells such as astrocytes. In our study, we observed that apoptosis in hUCBSC-treated nude mice tumor brains was carried out by the upregulation of TRAIL and TNF-α. TRAIL belongs to the TNF cytokine family and is capable of inducing apoptosis in a variety of cancer cells, while producing negligible effects on normal cells [55]. Our results show that hUCBSC are able to activate both apoptotic mechanisms mediated by caspase-3 as well as TRAIL, which ultimately inhibits the growth of the tumors by inducing apoptosis. Finally, the localization of Smac/DIABLO in the nucleus of the hUCBSC-treated brain sections is a clear indication of apoptosis taking place in the treated brains.

In conclusion, the growth retardation of glioblastoma cells treated with hUCBSC is not only due to the induction of apoptosis via caspase activation but also due to the downregulation of Akt and the involvement of mitochondrial apoptotic factors. Targeting XIAP by using hUCBSC might be an effective new strategy for the potential therapy of human gliomas.

## Materials and Methods

### Ethics Statement

After obtaining informed consent, human umbilical cord blood was collected from healthy volunteers according to a protocol approved by the Peoria Institutional Review Board, Peoria, IL, USA. The consent was written and approved. The approved protocol number is 06-014, dated December 10, 2009. The Institutional Animal Care and Use Committee of the University Of Illinois College Of Medicine at Peoria, Peoria, IL, USA approved all surgical interventions and post-operative animal care. The consent was written and approved. The approved protocol number is 851, dated November 20, 2009.

### Cell Cultures

Two high-grade human glioma cell lines SNB19 and U251 and two xenograft cell lines 4910 and 5310 were used for this study. SNB19 and U251 cells lines were obtained from American Type Culture Collection (ATCC, Manassas, VA). Two xenograft cell lines (4910 and 5310) were kindly provided by Dr. David James at University of California, San Francisco. SNB19 and U251 cells were grown in DMEM supplemented with 10% fetal bovine serum (FBS) (Hyclone, Logan, UT) and 1% penicillin-streptomycin (Invitrogen, Carlsbad, CA). Xenograft cell lines 4910 and 5310 were grown in RPMI-1640 medium supplemented with 10% FBS and 1% penicillin-streptomycin. For hUCBSC, after obtaining informed consent, human umbilical cord blood was collected from healthy volunteers according to a protocol approved by the Institutional Review Board. Cord blood was processed as described previously by sequential Ficoll density gradient purification [56]. Next, we selected cells using CD29 and CD81 markers as described previously. The nucleated cells were grown in Mesencult medium (Stem cell Technologies, Vancouver, Canada) supplemented with 20% FBS, 1% penicillin-streptomycin and plated in 100 mm culture dishes. All the cells were grown at 37°C in an incubator with 5% CO_2_ atmosphere. Human astrocytes were purchased from Sciencell Research Laboratories (Carlsbad, CA) and were grown in astrocyte medium supplemented with 2% FBS, 1% penicillin-streptomycin and 1% astrocyte growth supplements (Sciencell Research Laboratories). For co-culture experiments, hUCBSC/astrocytes and glioma cells were cultured at a ratio of 1∶4. Co-cultures of hUCBSC and SNB19, hUCBSC and U251 were grown in DMEM; co-cultures of hUCBSC and 4910, hUCBSC and 5310 were grown in RPMI-1640; similarly co-cultures of astrocytes and SNB19, astrocytes and U251 were grown in DMEM; co-cultures of astrocytes and 4910, astrocytes and 5310 were grown in RPMI-1640.

For co-cultures with astrocytes, DMEM and RPMI-1640 were supplemented with 1% astrocyte growth supplements. We observed that 1% astrocyte growth supplements did not show any effect on the growth of glioma cells (SNB19 and U251) and xenograft cells (4910 and 5310), when they were grown alone.

### Evaluation of cell death by LDH assay

The cytotoxic effect of hUCBSC on glioma cells was evaluated by measuring lactate dehydrogenase (LDH) activity released in the media 72 h after co-culture with hUCBSC using the CytoTox96 non-radioactive assay (Promega, Madison, WI). The experiment was performed as per the manufacturer's instructions and results were quantified by measuring wavelength absorbance at 490 nm. The experiment was performed three times (n = 3) with 3 wells per condition each time.

### Measurement of cell proliferation by MTT assay

We examined cell proliferation in single cultures and co-cultures of glioma cells with hUCBSC. The cultured glioma cells and co-cultures with hUCBSC (100 μL medium) were plated in 96-well microtiter plates at a final concentration of 0.5×10^5^ cells/well. The MTT solution (5 mg/mL) was prepared in DMEM/RPMI medium, and 10 μL were added to each well after treatment period as described previously (56). Absorbance of converted dye was measured at a wavelength of 570 nm with background subtracted at 630 nm (Bio-Rad microplate reader). Data were presented as percentage of MTT reduction as compared to control cells. The experiment was performed three times (n = 3) with 3 wells per condition each time.

### RNA extraction and reverse transcription-based PCR

All primer sequences were determined using established human GenBank sequences. Primer sequences were designed using Primer3 (v.0.4.0) software. Total RNA was isolated from control and hUCBSC-treated mice brains using Rneasy kit (Qiagen, Valencia, CA) and quantity were determined by A_260_ measurement. Total RNA was reverse transcribed into first strand cDNA using Transcriptor First Strand cDNA Synthesis Kit (Roche, Indianapolis, IN). Each cDNA was tested by running PCR using GAPDH or β-actin primer as a control for assessing PCR efficiency and for subsequent analysis by 2% agarose gel electrophoresis. PCR amplification was performed using the primer sets, amplified by 35 cycles (94°C, 1 min; 60°C, 1 min; 72°C, 1 min) of PCR using 20 pM of specific primers.

*Primers used for PCR*

XIAP:

Sense: 5′ggccagactatgcccattta3′

Antisense: 5′cgaagaagcagttgggaaa3′

β-Actin:

Sense: 5′gtcgtaccactggcattgt3′

Antisense: 5′cagctgtggtggtgaagct3′

### Immunoblot analysis of proteins

Single and co-cultures of glioma cells, siXIAP transfected cells or nude mice brain tissues were harvested and homogenized in four volumes of homogenization buffer as described previously [56]. Samples (40–50 µg of total protein/well) were subjected to 10–14% SDS-PAGE and transferred onto nitrocellulose membranes. The following antibodies were used for Western blot analysis: mouse anti-XIAP (1∶5000; BD Biosciences, Franklin Lakes, New Jersey), rabbit anti-AKT (1∶1000; Cell Signaling Technology Inc.), mouse anti-phospho-AKT (Ser^473^) (1∶1000; Cell Signaling Technology Inc.), mouse anti-Bax (1∶200; Santa Cruz Biotechnology), mouse anti-Bad (1∶200; Santa Cruz Biotechnology), rabbit anti-Bcl-2 (1∶200; Santa Cruz Biotechnology), rabbit anti-cleaved caspase 3 antibody (1∶1000; Abcam), rabbit anti-TNF-α (1∶1000; Cell Signaling), rabbit anti-TRAIL (1∶1000; Abcam), and rabbit anti-PARP (1∶1000; Cell Signaling Technology Inc.). Immunoreactive bands were visualized using chemiluminescence ECL Western blotting detection reagents (Amersham, Piscataway, NJ). The reaction was detected using Hyperfilm-MP autoradiography film (Amersham, Piscataway, NJ). Immunoblots were stripped and redeveloped with GAPDH antibody [mouse anti-GAPDH (1∶1000; Santa Cruz Biotechnology)] to ensure equal loading levels. Experiments were performed in triplicate. Values for treated and untreated samples were compared using one-way ANOVA. A *p* value of <0.05 was considered significant.

### Measurement of apoptosis and mitochondrial membrane potential

Apoptosis and the integrity of the mitochondrial membrane potential (Ψm) were evaluated with the Vybrant Apoptosis Assay Kit (Cat. No. V35116, Invitrogen, Carlsbad, CA). Apoptosis was induced by co-culturing of glioma cells with hUCBSC for 3 days. The concentration of the cells was adjusted to 5×10^6^ cells/mL in culture medium. To 1 mL of cells, 4 µL of 10 µM MitoTracker® Red working solution was added and stained for 30 min at 37°C in an atmosphere of 5% CO_2_. After incubation, cells were washed with PBS and resuspended in 100 µL of 1× Annexin-binding buffer. To this, 5 µL of Alexa Fluor® 488 Annexin V was added and the cells were incubated at room temperature for 15 minutes. After the incubation period, 400 µL 1× Annexin-binding buffer was added, mixed gently and the samples were placed on ice. The cells were analyzed by flow cytometry, measuring the fluorescence emission at 530 nm and 585 nm using BD FACSCalibur (BD Biosciences). In a similar manner, siXIAP transfected cells were processed for the measurement of apoptosis and mitochondrial membrane potential.

### Determination of activity of caspase-3 and caspase-9

Caspase-3 and caspase-9 activity of cells were measured using kits purchased from Millipore (Kankakee, IL). Control and treated cells (co-cultures or siXIAP-transfected cells) were used for this study. Treated and untreated cells were homogenized in 1× cell lysis buffer and the homogenates were centrifuged at 10,000xg for 5 min at 4°C in a microcentrifuge. Using the 96-well plate micro assay method, the supernatants were analyzed for caspase-3 or caspase-9 activity levels. In a final volume of 100 µL, supernatants (50 µg) of each test sample were incubated for 60 min at 37°C in the working solution containing Ac-DEVD-pNA, a synthetic caspase-3 substrate. Absorbance was read at 405 nm in an ELISA plate reader after a period of 60 min. Ac-DEVD-CHO inhibitor was used for inhibitor studies. For experiments with inhibitor, the samples were pre-incubated with Ac-DEVD-CHO inhibitor (0.1 µM) for 10 minutes at room temperature before adding caspase-3 substrate solution. Caspase-3 activity was calculated as micromolar per gram of cells using a p-nitroaniline calibration curve. The data were plotted as A_405_ versus time for each sample and activity was calculated as pmol/min. In a similar manner, cells were also processed for caspase-9 activity using Caspase-9 Substrate (Ac-LEHD-pNA) and Caspase-9 Inhibitor (Ac-LEHD-CHO). For experiments with inhibitor, the samples were pre-incubated with Ac-LEHD-CHO inhibitor (0.1 µM) for 10 minutes at room temperature before adding caspase-9 substrate solution. The experiments were repeated 3 times.

### Intracranial tumor growth inhibition

The Institutional Animal Care and Use Committee of the University Of Illinois College Of Medicine at Peoria approved all surgical interventions and post-operative animal care. For the intracerebral tumor model, U251 (1×10^6^ cells) and 5310 (8×10^5^ cells) tumor cells were intracerebrally injected into the right side of the brain of the nude mice as described previously [57]. Seven days after tumor implantation, the mice were injected with hUCBSC towards the left side of the brain. The ratio of the hUCBSC to glioma cells was maintained at 1∶4. Three weeks after tumor inoculation, six mice from each group were sacrificed by cardiac perfusion with 4% formaldehyde in PBS, their brains were removed, and paraffin sections were prepared. Sections were stained with Hematoxylin & Eosin (H&E) to visualize tumor cells and to examine tumor volume. The sections were blindly reviewed by a neuropathologist and scored semiquantitatively for tumor size. Whole-mount images of brains were also taken to determine infiltrative tumor morphology. The average tumor area per section integrated to the number of sections where the tumor was visible was used to calculate tumor size and compared between controls and treated groups. Immunoblot analyses and RT-PCR were done on fresh brain tissues.

### Immunohistochemical analysis

Brains of control and hUCBSC-treated mice were fixed in formaldehyde and embedded in paraffin as per standard protocols. Sections were deparaffinized and blocked in 1% BSA in PBS for 1 h, and the sections were subsequently transferred to primary antibody diluted in 10% normal goat serum (1∶100). Sections were allowed to incubate in the primary antibody solution overnight at 4°C in a humidified chamber. Sections were then washed in 1% BSA in PBS and placed in a solution with the appropriate secondary antibody. The sections were incubated with the secondary antibody for 1 h and visualized using a light/confocal microscope. Transmitted light images were obtained after H&E staining as per standard protocol to visualize the morphology of the sections. Negative controls were maintained without primary antibody or by using IgG fraction.

### *In situ* terminal-deoxy-transferase mediated dUTP nick end labeling (TUNEL) assay

A TUNEL apoptosis detection kit (Roche) was used for DNA fragmentation fluorescence staining according to the manufacturer's protocol. Briefly, glioma cells co-cultured with hUCBSC or transfected with either siXIAP or scrambled vector (SV) or brain sections were used for this study. Seventy-two hours after co-culture or transfection, cells were fixed with 4% paraformaldehyde in 0.1 M phosphate buffer (pH 7.4). Next, cells were incubated with a reaction mix containing biotin-dUTP and terminal deoxynucleotidyl transferase for 60 min. Fluorescein-conjugated avidin was applied to the samples, which were then incubated in the dark for 30 min. Positively stained fluorescein-labeled cells were visualized and photographed using fluorescence microscopy. For TUNEL assay of mice brain sections, a similar procedure was followed after deparaffinization of the sections.

### Construction of shRNA-expressing plasmid and transfections

For this study, pSilencer™ 4.1-CMV neo vector (Ambion, Austin, TX) was used in the construction of the shRNA-expressing vector. The Rat XIAP target sequence AACTGGACAGGTTGTAGATAT was used for the shRNA sequence. Inverted repeat sequences were synthesized for XIAP. The inverted repeats were laterally symmetrical, making them self-complimentary with a 9-bp mismatch in the loop region. This 9-bp mismatch would aid in the loop formation of the shRNA. Oligonucleotides were heated in a boiling water bath in 6× SSC for 5 min and self-annealed by slow cooling to room temperature. The resulting annealed oligonucleotides were ligated to pSilencer at the BamHI and HindIII sites. Glioma cells at 60–70% confluency in 100 mm tissue culture plates were transfected with 10 µg of siRNA-expressing plasmid constructs [scrambled vector (SV) or siXIAP] using Fugene-HD as per the manufacturer's instructions (Roche). Following transfection, after 60 to 72 h depending on the cell line, cell lysates were assessed for expression levels of different proteins using western blot analysis as per standard protocol.

### Fluorescent *in situ* hybridization (FISH) analysis

Serial 5 µm cross-sections were prepared on a cryostat, thaw mounted on slides coated with 3-aminopropyltriethoxysilane (Sigma, St. Louis, MO) and stored frozen until they were used for *in situ* hybridization. Oligonucleotide antisense sequences with a length of 48 bases were used as probes for the following genes:

XIAP Sense: AATGCTTTTGTTGTGGTGGAAAACTGAAAAATTGGGAACCCTGTGA

XIAP Antisense: TCACAGGGTTCCCAATTTTTCAGTTTTCCACCACAACAAAAGCATT

The oligonucleotides were labeled with FITC at 3′ ends (Sigma-Genosys, The Woodlands, TX) and were processed for FISH analysis as described previously [58]. Briefly, slides were post-fixed with 4% formaldehyde in PBS (pH 7.4) for 10 min, acetylated (0.25% acetic anhydride in 0.1 M triethanolamine HCl, pH 8) for 10 min, and dehydrated with graded alcohols and chloroform. They were then incubated overnight at 37°C with hybridization buffer containing 200 ng/mL of each oligonucleotide probe. The next day, slides were washed sequentially with 2× SSC (0.15 M NaCl, and 15 mM sodium citrate, pH 7.0) for 5 min at room temperature, 0.2× SSC (1 h at 72°C in shaking water bath) and 0.2× SSC (5 min at room temperature) and then allowed for detection of fluorescent-labeled probes using ELF 97 mRNA *in situ* hybridization kit (Invitrogen, Carlsbad, CA). Finally, the slides were counterstained with Hoechst 333342 (for visualization of cell nuclei) and mounted using mounting medium. Visualization of FISH signal was done with a fluorescence microscope (IX71 Olympus) and/or a confocal microscope (Olympus Fluoview). Sections stained with sense probes served as controls, which do not show any signal.

### Statistical analysis

Quantitative data from cell counts, Western blot analysis, and other assays were evaluated for statistical significance using one-way analysis of variance (ANOVA). Data for each treatment group were represented as mean ± SEM and compared with other groups for significance by one-way ANOVA followed by Bonferroni's post hoc test (multiple comparison tests) using Graph Pad Prism version 3.02, a statistical software package. Results were considered statistically significant at *p* less than 0.05.

## Supporting Information

Figure S1 Growth inhibition of glioma cells by siXIAP. (A) MTT assay of SV and siXIAP treatments of glioma cells. (B) Cytotoxicity assay based on cytosolic LDH assay. (C) FACS analysis results of glioma cells showing apoptotic cells as measured by Annexin V. Each experiment was repeated 3 times. Error bars indicate ±SEM. * significant at p<0.05.
(5.45 MB TIF)

Figure S2 Immunoblot analysis of proteins with cell lysates of siXIAP treatments. 40 µg of proteins were loaded onto 12–14% gels, transferred onto nitrocellulose membranes, and probed with respective antibodies. Immunoreactive bands were visualized using chemiluminescence ECL Western blotting detection reagents and the reaction was detected using Hyperfilm-MP autoradiography film. Each experiment was repeated 3 times.
(5.64 MB TIF)

Figure S3 Immunoblot analysis of proteins with cell lysates of hUCBSC treatments at different time points. 40 µg of proteins were loaded onto 12–14% gels, transferred onto nitrocellulose membranes, and probed with respective antibodies. Immunoreactive bands were visualized using chemiluminescence ECL Western blotting detection reagents and the reaction was detected using Hyperfilm-MP autoradiography film. Each experiment was repeated 3 times.
(5.16 MB TIF)

Figure S4 Activity of caspases in siXIAP treatments. (A) Caspase-3 activity in single and siXIAP transfected glioma cells. (B) Caspase-9 activity in single and siXIAP transfected glioma cells. Both these assays were done as described in Materials and Methods. C3I  =  Caspase-3 Inhibitor (Ac-DEVD-CHO); C9I  =  Caspase-9 inhibitor (Ac-LEHD-CHO). Each experiment was repeated 3 times. Error bars indicate ±SEM. *Significant at p<0.05.
(8.74 MB TIF)
